# Effects of Sevoflurane Laryngeal Mask Inhalation Combined with Intravenous Anesthesia on Perioperative Stress and Myocardial Injury in Elderly Patients with Acute Cholecystitis and Coronary Heart Disease

**DOI:** 10.1155/2022/6482491

**Published:** 2022-11-12

**Authors:** Wei Jin, Xiaoxing Shen, Hongxu Jin

**Affiliations:** Department of Anesthesiology, Harrison International Peace Hospital, Hebei Medical University, Hengshui 053000, Hebei, China

## Abstract

Surgery is the first choice for the treatment of acute cholecystitis. To ensure the curative effect of surgery, laparoscopic anesthesia should be characterized by rapid induction, good analgesic effect, and rapid postoperative sobriety. With the aggravation of an aging population, acute cholecystitis combined with coronary heart disease is more common in the elderly. The selection of anesthesia protocols for these patients has become a hot topic in research. In this study, we selected 72 elderly patients with acute cholecystitis combined with coronary heart disease who were treated in our hospital from January 2019 to January 2022 to explore the effects of sevoflurane laryngeal mask inhalation combined with intravenous anesthesia on perioperative stress and myocardial injury in elderly patients with acute cholecystitis combined with coronary heart disease, in order to provide a scientific basis for the formulation of a surgical plan for elderly patients with acute cholecystitis combined with coronary heart disease.

## 1. Introduction

Coronary heart disease is a multiple cardiovascular disease in the middle-aged and elderly people. Patients with coronary heart disease are often older and suffer from other diseases at the same time. Acute cholecystitis is one of them. Acute cholecystitis is inflammation of the gallbladder caused by obstruction of the cystic duct and bacterial invasion, and it includes acute calculous cholecystitis and acute acalculous cholecystitis [1]. Acute cholecystitis is mainly manifested as epigastric pain radiating to the right shoulder and back. Clinically, the disease develops very rapidly. With the development of the disease, patients may have unbearable pain, restlessness, intolerance of cold and high fever, and even life-threatening conditions in severe cases [2]. Early surgical intervention is the key to saving patients with acute cholecystitis [3]. Anesthesia is the most essential part of surgery. The condition of elderly patients with cholecystitis combined with coronary heart disease is often complex, and the selection of an anesthesia scheme for such patients is also difficult.

At present, the commonly used clinical anesthesia methods are divided into intravenous general anesthesia and inhalation anesthesia. And with the rapid development of anesthesia technology and equipment, a variety of new anesthesia methods have been gradually applied in clinical practice to ensure that surgical complications caused by respiratory problems are minimized. The laryngeal mask is an artificial airway placed in the throat cavity, using a balloon to seal the esophagus and throat cavity, and ventilating through the laryngeal cavity, avoiding tracheal intubation, but it is more effective than using a mask. It has been clinically proven for more than two decades for its remarkable effect in resolving or managing common and difficult airways [4]. Sevoflurane does not need intravenous injection and can produce obvious anesthesia effect on human body after being inhaled through the respiratory tract and has the advantages of quick effect, quick recovery, good controllability, and a small toxic side effect. In recent years, sevoflurane has become the most widely used inhalation anesthetic in the global anesthesiology community [5]. However, few studies have reported its application value in elderly patients with acute cholecystitis combined with coronary heart disease. Therefore, this study investigated the effect of sevoflurane laryngeal mask inhalation combined with intravenous anesthesia on perioperative stress and myocardial injury in elderly patients with acute cholecystitis complicated by coronary heart disease. It aims to provide a better basis for the clinical treatment of such patients.

## 2. Materials and Methods

### 2.1. General Information

A total of 72 elderly patients with acute cholecystitis complicated by coronary heart disease who visited our hospital from January 2019 to January 2022 were selected as the research objects. The patients were divided into an observation group and a control group according to the random number table method, with 36 cases in each group. There were 14 males and 22 females in the control group ranging in age from 61 to 82 years mean age: 71.54 ± 5.27 years; and there were 33 cases of acute calculous cholecystitis, 3 cases of acute acalculous cholecystitis, 12 cases of arrhythmia, 11 cases of hypertension, and 4 cases of diabetes. There were 15 males and 21 females in the observation group. Their age ranged from 61 to 85 years, with an average of 73.04 6.02 years. And there were 33 cases of acute calculous cholecystitis; 3 cases of acute acalculous cholecystitis; 10 cases of combined arrhythmia; 10 cases of hypertension; and 3 cases of diabetes. There was no significant difference in the basic data between the two groups (*P* > 0.05). The study was reviewed and approved by the Hospital Ethics Committee, and the patient and his/her family were aware of the study and signed an informed consent form.

### 2.2. Inclusion Criteria

① Meet the relevant diagnostic criteria for acute cholecystitis and coronary heart disease [6, 7]; ② age more than 60 years old; ③ ASA grade I～III; and ④ comply with the indications of laparoscopic surgery, no contraindications.

### 2.3. Exclusion Criteria

① Patients with coagulation dysfunction; ② patients with liver and kidney damage; ③ patients with other heart diseases other than related diseases; ④ patients with mental disorders; ⑤ patients with respiratory system-related diseases; and ⑥ those who have severe allergies to the drugs used in this study.

### 2.4. Methods

Both groups underwent an elective laparoscopic cholecystectomy. The rats were deprived of food for 8 h and 4 h before operation. The intramuscular injection of 0.5 mg atropine sulfate injection (Wanbangde Pharmaceutical Group Co., Ltd., H13022141) and 0.1 g benzene was performed. The barbital sodium injection (Tianjin Jinyao Pharmaceutical Co., Ltd., recognized by TCM as H12020381) was performed 0.5 h before anesthesia. The upper limb veins were opened for monitoring blood pressure, heart rate, electrocardiogram and other vital signs.

#### 2.4.1. Control Group

The oxygen saturation of blood oxygen was maintained at 98% with mask oxygen inhalation. Propofol injection (AstraZeneca S.p.A., Italy, import drug registration number: H20080473) compound remifentanil hydrochloride for injection (Yichang Renfu Pharmaceutical Co., Ltd. Company, Sinopharm Zhunzi H20030197) anesthesia, intravenous injection of propofol injection 2 *μ*g/kg and remifentanil hydrochloride 200 *μ*g/kg for anesthesia induction, after the patient lost consciousness, intravenous injection of 0.1 mg/kg vitamin for injection. Curium bromide (Zhejiang Xianju Pharmaceutical Co., Ltd., approved by Chinese medicine H19991172), tracheal intubation after 5 minutes, mechanical ventilation (tidal volume 8–10 mL/kg) to control respiratory rate 12 times/min, propofol maintenance anesthesia was performed at 0.2 mg/(kg·min), and propofol was discontinued after the operation.

### 2.5. Observation Group

The oxygen saturation of blood oxygen was maintained at 98% by mask oxygen inhalation and sevoflurane for inhalation (Shanghai Baxter Medical Products Co., Ltd., Imported Drug Registration Certificate No.: H20110142) compound remifentanil hydrochloride for injection (Yichang Renfu Pharmaceutical Co., Ltd., responsible company, Chinese medicine Zhunzi H20030197) during intravenous inhalation anesthesia. The target-controlled infusion of remifentanil, with a target plasma concentration of 3 ng/mL was performed. The oxygen switch was turned on and was set the flow rate to 5 L/min. Then the sevoflurane evaporator was opened until 0 patient lost consciousness, and the laryngeal mask was placed. After that, 0.1 mg/kg vecuronium bromide for injection was given intravenously (Zhejiang Xianju Pharmaceutical Co., Ltd.). Company, GuoYaoZhunZi H19991172), mechanical ventilation (tidal volume 8–10 mL/kg) control the respiratory rate of 12 times/min, remifentanil maintain a constant target concentration, sevoflurane maintain anesthesia inhalation concentration of 0.8–1.5%, sevoflurane and remifentanil stopped after surgery.

### 2.6. Observation Indicators

#### 2.6.1. Comparison of Anesthesia Effects

The orientation recovery time, spontaneous breathing recovery time, eye opening time, and speech response time of the two groups were observed and recorded.

#### 2.6.2. Comparison of Perioperative Stress

1. The levels of hemodynamic indexes, including mean arterial pressure (MAP) and heart rate (HR), were observed and recorded before anesthesia (T0), 1 min after intubation (T1), during skin incision (T2), 5 min after pneumoperitoneum (T3), and after surgery (T4) in the two groups.
2. 5 mL of fasting venous blood was collected from both groups before operation, immediately after operation, 6 hours after operation, and 12 hours after operation. The blood was centrifuged at 3000 r/min for 10 minutes, separated and collected the upper serum part, which was divided into two parts and stored in −80°C refrigerator to be tested. Stress response indicators (cortisol (Cor), C-reactive protein (CRP)) were detected using ELISA kits (Shanghai Qiyan Biotechnology Co., Ltd.).

#### 2.6.3. Comparison of Myocardial Injury

The supernatant serum collected in 1.4.2 was used for testing. The indicators of myocardial injury, creatine kinase isoenzyme MB (CK-MB), and cardiotrophin I (cTnI), were detected by ELISA. The kits were purchased from Shanghai Qiyan Biotechnology Co., Ltd.

### 2.7. Statistical Methods

All counting and measurement data were input into SPSS 22.0 software for statistical data analysis, and Shapiro-Wilk was used for a normality test for measurement data. The data that meet the normal distribution are expressed in the form of (±S), an independent *t*-test is used, and the comparison of multiple time points within the group uses the analysis of variance of repeated measures data. Enumeration data were expressed as number of cases or rate, and differences between groups were compared using *χ*^2^ test. A statistical value *P* < 0.05 indicates statistical significance.

## 3. Results

### 3.1. Comparison of Indexes Related to Anesthesia Effect Between the Two Groups

The orientation recovery time, spontaneous breathing recovery time, eye opening time, and speech response time of the observation group were shorter than those of the control group (*P* < 0.05). As shown in Figure 1 and Table 1.

### 3.2. Comparison of Perioperative Hemodynamic Indexes between the Two Groups

At T0, there was no significant difference in the levels of MAP and HR between the observation group and the control group (*P* > 0.05). From T1 to T4, the levels of MAP and HR in the two groups first decreased and then increased (*P* < 0.05), and the observation group was higher than the control group (*P* < 0.05) as shown in Figures 1 and 2 and Table 2.

### 3.3. Comparison of Perioperative Serum Stress Response Indexes between the Two Groups

There was no significant difference in serum Cor and CRP levels between the observation group and the control group before operation (*P* > 0.05); Immediately after operation, the levels of serum Cor and CRP in the two groups were increased, and decreased at 6 hours and 12 hours after operation (*P* < 0.05), and the observation group was lower than the control group (*P* < 0.05) as shown in Figure 3 and Table 3.

### 3.4. Comparison of Perioperative Serum Myocardial Injury Indexes between the Two Groups

Before operation and immediately after operation, there was no significant difference in serum CK-MB and cTnI levels between the observation group and the control group (*P* > 0.05); The levels of serum CK-MB and cTnI in the two groups increased at 6 hours and 12 hours after operation (*P* < 0.05), but the observation group was lower than the control group (*P* < 0.05) as shown in Figure 4 and Table 4.

## 4. Discussions

Acute cholecystitis is a digestive tract emergency that can occur in any age group. Surgery is one of the main treatment methods for acute cholecystitis, but the physiological reserve ability of elderly patients is poor due to their own physical condition and combined with coronary heart disease. Therefore, it is necessary to comprehensively formulate the surgical plan according to the actual situation and physical quality of such patients, especially to select the appropriate anesthesia plan [8].

Relevant studies reported that different anesthesia methods may cause different anesthesia effects and stress responses in elderly patients, which may have a certain impact on the successful completion of surgery [9]. In this study, the recovery time of orientation, spontaneous breathing, eye opening, and speech response time in the observation group were shorter than those in the control group, suggesting that sevoflurane laryngeal mask inhalation combined with intravenous anesthesia is effective for elderly patients with acute cholecystitis complicated by coronary heart disease. The effect of perioperative anesthesia is good, and it will not cause respiratory depression caused by excessive anesthesia. Inhalation anesthesia is a commonly used anesthesia method in clinic. Anesthesia by respiratory inhalation reduces drug metabolism and decomposition in the body, allowing most of it to be excreted directly from the lungs. Therefore, inhalation anesthesia is easy to control and relatively safe and effective. Sevoflurane is a surgical anesthetic that is widely used in clinical practice, which was more convenient to used. Its physical properties were superior to those of the existing human anesthetics, and the blood/air fraction coefficient was only 0.59. Due to rapid induction and small tissue uptake, the patient recovered quickly after surgery. Studies have confirmed that patients under sevoflurane anesthesia generally recover less than 10 minutes after drug discontinuation, and patients have no symptoms of falling asleep again after waking up, and there are obvious complications such as nausea and vomiting, dizziness, headache, cough, throat and bronchospasm, edema, and other complications [10, 11].

Traditional anesthesia requires endotracheal intubation, and there are many receptors in the throat. Direct endotracheal intubation can cause intense stimulation, leading to arousal of sympathetic nervous system and aggravation of cardiovascular stress response, which may aggravate coronary heart disease in patients [12]. The results of this study found that, at T1-T4, the levels of MAP and HR in the two groups first decreased and then increased, and the observation group was higher than the control group. The study by Kannojiya et al. [13] reported that the application of a laryngeal mask in pediatric laparoscopic surgery has less effect on the hemodynamic parameters of patients and fewer postoperative complications. Combined with the above reports, this study believe that sevoflurane laryngeal mask inhalation combined with intravenous anesthesia has a stable effect on perioperative hemodynamic parameters of elderly patients with acute cholecystitis combined with coronary heart disease and can reduce surgical stress. The stress response indexes of the two groups were further analyzed, and it was also found that the serum Cor and CRP levels of the two groups increased at 6 h and 12 h after the operation, but the observation group was lower than the control group. Cor and CRP can be used as indicators of decreased surgical stress response after laparoscopic surgery [14, 15]. The reason may be that, compared with tracheal intubation, the laryngeal mask does not need to use instruments to expose the glottis, the throat irritation is small, so it does not enter the trachea, it has no irritation to the tracheal mucosa, and its hemodynamics are less affected.

Relevant research have reported that for the elderly patients with coronary heart disease, the use of irritating anesthesia methods such as tracheal intubation during the operation easily induces serious cardiovascular complications, such as such as increased blood pressure and arrhythmia [16]. The results of this study showed that the serum levels of CK-MB and cTnI in the two groups were increased at 6 h and 12 h after the operation, but the observation group was lower than the control group. Zhang et al. [17] found that sevoflurane inhalation anesthesia can effectively maintain perioperative hemodynamic stability in elderly patients with coronary heart disease and has a certain myocardial protection effect. The analysis of the reason may be related to the efficacy of sevoflurane in increasing the opening of intracellular ATP-sensitive potassium channels, increasing cardiac output, and reducing coronary neutrophil adhesion [18].

In conclusion, the application of sevoflurane laryngeal mask inhalation combined with intravenous anesthesia in elderly patients with acute cholecystitis complicated by coronary heart disease can relieve the perioperative stress response, ensure stable hemodynamics in the perioperative period, and promote rapid and stable recovery. And it will not aggravate the myocardial injury of patients, improving the safety of anesthesia. However, there are still some deficiencies in this study. For example, it is a single-center study with a small number of samples, and there may be some data biases. In the later stage, further multi-center and large-sample clinical trials are needed for in-depth research.

## Figures and Tables

**Figure 1:** Level distribution of indexes related to the anesthesia effect in two groups (Note. (a) Level distribution of indexes related to anesthesia effect in the control group; (b) Level distribution of indexes related to anesthesia effect in the observation group).

**Figure 2:** Comparison of perioperative hemodynamic indexes between the two groups (Note. (a) Comparison of perioperative MAP levels between the observation group and the control group; (b) comparison of HR levels between the observation group and the control group in the perioperative period).

**Figure 3:** Comparison of perioperative serum stress response indexes between the two groups (Note. (a) Comparison of perioperative Cor levels between observation group and control group; (b) comparison of perioperative CRP levels between observation group and control group).

**Figure 4:** Comparison of perioperative serum myocardial injury indexes between the two groups (Note. (a) Comparison of perioperative CK-MB levels between observation group and control group; (b) comparison of perioperative cTnI levels between the observation group and control group).

**Table 1:** The indexes related to the anesthesia effect of the two groups ($\bar{x}$ ± *s*, min).

Group	*n*	Orientation recovery time	Spontaneous breathing recovery time	Eye opening time	Verbal response time
Control group	36	16.23 ± 1.16	8.63 ± 0.74	13.32 ± 2.16	19.34 ± 1.59
Observation group	36	12.72 ± 1.58	6.17 ± 0.51	9.05 ± 1.74	15.60 ± 1.58
*t*		10.744	16.423	9.237	10.011
*P*		<0.001	<0.001	<0.001	<0.001

**Table 2:** Comparison of perioperative hemodynamic indexes between the two groups ($\bar{x}$ ± *s*).

Time	MAP (mm·Hg)		HR (beats/min)	
	Control group (*n* = 36)	Observation group (*n* = 36)	Control group (*n* = 36)	Observation group (*n* = 36)
T0	104.00 ± 7.05	104.08 ± 5.30	86.75 ± 7.83	85.39 ± 6.89
T1	86.50 ± 7.50^*∗*^	91.94 ± 5.70^*∗*^^#^	69.86 ± 6.69^*∗*^	73.83 ± 6.44^*∗*^^#^
T2	90.22 ± 6.53^*∗*^	94.11 ± 6.05^*∗*^^#^	73.97 ± 7.57^*∗*^	78.31 ± 6.36^*∗*^^#^
T3	95.14 ± 7.22^*∗*^	98.56 ± 6.10^*∗*^^#^	77.58 ± 6.75^*∗*^	81.42 ± 7.20^*∗*^^#^
T4	99.61 ± 7.88^*∗*^	104.25 ± 7.57^#^	80.89 ± 7.07^*∗*^	84.17 ± 5.10^#^

*F*_group_/*P*_group_	4.327/0.045		4.159/0.049	
*F*_time_/*P*_time_	64.683/<0.001		41.104/<0.001	
*F*_mutual_/*P*_mutual_	55.444/<0.001		56.374/<0.001	

Note. Compared with T0, ^*∗*^*P* < 0.05; compared with control group, ^#^*P* < 0.05.

**Table 3:** Comparison of perioperative serum stress response indexes between the two groups ($\bar{x}$ ± *s*).

Time	Cor (*μ*g/L)		CRP (mg/L)	
	Control group (*n* = 36)	Observation group (*n* = 36)	Control group (*n* = 36)	Observation group (*n* = 36)
Preoperative	256.44 ± 65.96	268.50 ± 47.80	27.51 ± 2.86	27.17 ± 4.33
Immediately after surgery	473.58 ± 59.58^*∗*^	372.14 ± 64.22^*∗*^^#^	55.46 ± 4.40^*∗*^	43.96 ± 6.35^*∗*^^#^
6 h after surgery	368.67 ± 56.59^*∗*^	324.03 ± 52.14^*∗*^^#^	43.13 ± 4.18^*∗*^	37.15 ± 4.96^*∗*^^#^
12 h after surgery	299.37 ± 50.78^*∗*^	265.07 ± 57.02^#^	35.06 ± 4.04^*∗*^	27.34 ± 4.80^#^

*F*_group_/*P*_group_	12.039/0.001		38.373/<0.001	
*F*_time_/*P*_time_	136.837/<0.001		316.524/<0.001	
*F*_mutual_/*P*_mutual_	287.283/<0.001		370.364/<0.001	

Note. Compared with preoperative, ^*∗*^*P* < 0.05; compared with control group, ^#^*P* < 0.05.

**Table 4:** Comparison of perioperative serum myocardial injury indexes between the two groups ($\bar{x}$ ± *s*).

Time	CK-MB (U/L)		cTnI (*μ*g/L)	
	Control group (*n* = 36)	Observation group (*n* = 36)	Control group (*n* = 36)	Observation group (*n* = 36)
Preoperative	1.05 ± 0.38	1.17 ± 0.36	0.30 ± 0.05	0.30 ± 0.04
Immediately after surgery	1.22 ± 0.35	1.20 ± 0.27	0.35 ± 0.12	0.33 ± 0.10
6 h after surgery	2.04 ± 0.77^*∗*^	1.68 ± 0.63^*∗*^^#^	0.92 ± 0.17^*∗*^	0.73 ± 0.14^*∗*^^#^
12 h after surgery	2.88 ± 0.86^*∗*^	2.23 ± 0.63^*∗*^^#^	1.34 ± 0.24^*∗*^	0.86 ± 0.07^*∗*^^#^

*F*_group_/*P*_group_	4.456/<0.042		35.336/<0.001	
*F*_time_/*P*_time_	432.741/<0.001		684.042/<0.001	
*F*_mutual_/*P*_mutual_	42.183/<0.001		191.062/<0.001	

Note. Compared with preoperative, ^*∗*^*P* < 0.05; compared with control group, ^#^*P* < 0.05.

## Data Availability

The data supporting the conclusion of this article will be available by the authors without undue reservation.
